# A Cloud-Based Machine Learning Approach to Reduce Noise in ECG Arrhythmias for Smart Healthcare Services

**DOI:** 10.1155/2022/3773883

**Published:** 2022-06-28

**Authors:** Paras Jain, Walaa F. Alsanie, Dulio Oseda Gago, Gilder Cieza Altamirano, Rafaél Artidoro Sandoval Núñez, Ali Rizwan, Simon Atuah Asakipaam

**Affiliations:** ^1^School of Computing Science and Engineering, VIT Bhopal University, Kothrikalan, Sehore, Madhya Pradesh 466114, India; ^2^Department of Clinical Laboratory Sciences, The Faculty of Applied Medical Sciences, Taif University, Taif, Saudi Arabia; ^3^Centre of Biomedical Sciences Research (CBSR), Deanship of Scientific Research, Taif University, Taif, Saudi Arabia; ^4^Universidad Nacional Mayor de San Marcos, Lima, Peru; ^5^Universidad Nacional Autónoma de Chota, Cajamarca, Peru; ^6^Department of Industrial Engineering, Faculty of Engineering, King Abdulaziz University, Jeddah 21589, Saudi Arabia; ^7^Tamale Technical University, Electrical and Electronics Engineering, Tamale, Ghana

## Abstract

ECG (electrocardiogram) identifies and traces targets and is commonly employed in cardiac disease detection. It is necessary for monitoring precise target trajectories. Estimations of ECG are nonlinear as the parameters TDEs (time delays) and Doppler shifts are computed on receipt of echoes where EKFs (extended Kalman filters) and electrocardiogram have not been examined for computations. ECG, certain times, results in poor accuracies and low SNRs (signal-to-noise ratios), especially while encountering complicated environments. This work proposes to track online filter performances while using optimization techniques to enhance outcomes with the removal of noise in the signal. The use of cost functions can assist state corrections while lowering costs. A new parameter is optimized using IMCEHOs (Improved Mutation Chaotic Elephant Herding Optimizations) by linearly approximating system nonlinearity where multi-iterative function (Optimized Iterative UKFs) predicts a target's unknown parameters. To obtain optimal solutions theoretically, multi-iterative function takes less iteration, resulting in shorter execution times. The proposed multi-iterative function provides numerical approximations, which are derivative-free implementations. Signals are updated in the cloud environment; the updates are received by the patients from home. The simulation evaluation results with estimators show better performances in terms of reduced NMSEs (normalized mean square errors), RMSEs (root mean squared errors), SNRs, variances, and better accuracies than current approaches. Machine learning algorithms have been used to predict the stages of heart disease, which is updated to the patient in the cloud environment. The proposed work has a 91.0% accuracy rate with an error rate of 0.05% by reducing noise levels.

## 1. Introduction

Target identifications/tracking, management of air traffic, and remote sensing are all common uses of ECG [1, 2] where transmitters send signal bursts and receivers receive dispersed versions of those signals. The scattering of signals is measured using TDEs and Doppler shifts in received signals, and the target's range and radial velocities are computed. These measurements are employed as measurements in ECG [3]. The fundamental concept of radars is similar to that of sound wave reflection. Radars detect and locate objects by using electromagnetic radiation bursts. Radars can be classified in a variety of ways, but categorized into eleven groups based on their functionality and primary characteristics [4].

Generic pulse radars play a prominent role in ECG where they emit a series of short-duration rectangular pulses in repeated patterns. Pulse radars can be divided into two categories, namely, radars with MTYIs (moving target indications) and radars with pulse Doppler. Both these types employ Doppler frequency shift, which works with incoming signals to find a moving target. The TDEs and Doppler shift are used to calculate measures such as range and radial velocity based on these two kinds. Difficulties in calculating TDEs between received signals of same transmitters are known as TDEs [5] where computing these parameters is critical for detecting targets with radar's transmitters. These received echoes are referenced with signals by the usage of filters to estimate TDEs and assure target recognitions.

New techniques in nonlinear estimation [6, 7] such as KLMSs (Kernel Least Mean Squares) have been developed that are efficient in estimating TDEs and Doppler shifts. Employing representational theorems and iterative estimation of nonlinearity between unknown parameters, RKHSs (Reproducing Kernel Hilbert's Spaces), are used to return signals while using KLMS estimators to estimate nonlinearity. The LMS approach in RKHSs is used to adaptively update the parameters that have been determined.

EKFs and UKFs are nonlinear estimators that are often employed in radar measurements and have been examined for tracking objects in radar measurements [8, 9]. Specific uses of synthetic aperture radars are as follows: Kalman filter's variant MCKFs (Modified Convolution Kernel Functions) [10] assessed parameters of returning LFMSs (Linear Frequency Modulated Signals) in certain cases [10]. TDEs and Doppler shifts in target tracing applications are estimated using EKFs and UKFs, which have not been studied in detail.

Rather than producing linear models, they approach nonlinear systems using first-order linearization, which results in linear models [11]. Because of their weak accuracy and stability in difficult situations with low SNRs and heavy-tailed clutters, they are unable to distinguish between targets with high certainty. In addition, improved EKFs and UKFs assess systems in their nonlinear true forms, which aids in the estimation of reliable parameter estimations even in challenging contexts [12]. It should be noted that the goal of IEKFs is to seek for superior linearization that is suitable for severe nonlinearities rather than to repair linearization errors directly [13]. They are a logical extension of EKFs, which combine NLSs (nonlinear least squares) with GNs to form a new class of EKFs known as IEKFs (Gaussian Newton).

Using optimization approaches, this work offers a multi-iterative function for monitoring filter performances in real time and striving to enhance them as much as possible. The usage of cost functions might help you keep track of state corrections and save money [14]. The optimization of a new parameter is carried out using MCEHOs, which approximate the nonlinearity of the system, and multi-iterative function, which estimates the unknown parameters of a target [16]. In order to optimise the underlying cost functions, a multi-iterative function technique based on the MCEHOs approach is used. As proven by the simulation findings, this research is able to obtain higher levels of accuracy.

## 2. Literature Review

Singh et al. [4] in their study proposed nonlinear estimations based on sparse KLMSs (Kernel Least Mean Squares). Their scheme used adaptive kernel width optimizations for reducing computational complexities and easier implementations [17]. The study used modulated and orthogonal frequency division multiplexed radar signals where Cramér–Rao lower bounds were constructed for their proposed estimations. Target ranges were estimated by Singh et al. [18] where unique iterative nonlinear KLMSs estimations were used. Their scheme when compared with FTs (Fourier Transforms) based estimation in simulations showed KLMSs converged with reduced MSEs. KLMSs have significant limitations in assessments on characteristics including kernel widths, step sizes, and dictionary threshold values, and when these parameters are run on specified ranges, they yield suitable values [19].

Kulikov and Kulikova [20] suggested accurate continuous-discrete EKFs based on ODEs (ordinary differential equations) with global error controls. They compared their proposed scheme with continuous-discrete cubature and UKFs using seven-dimensional radar tracking where aeroplanes made coordinated turns [21]. The study proved the worthiness of nonlinear filtering techniques in their tests by using them for actual target tracking; however, their accurate continuous-discrete EKFs were found to be versatile and resilient in their tests [22]. It could successfully address air traffic control situations for diverse data and variety of sample times without any manual adjustments.

Gu et al. [23] suggested multicomponent LFMS parameter estimations based on MCKFs. The suggested scheme was quicker as there were no searching operations, reduced external influences, and lowered computing burdens [24]. Furthermore, it was resistant to additive noises. Their suggested strategy was supported by simulated and real-world data. On the other hand, EKFs and UKFs have not been used to estimate the TDEs and Doppler shift for target tracking.

For global optimization issues, Ibrahim et al. [25] presented SKFs (Simulated Kalman Filters), a population-based metaheuristic optimization, based on Kalman filter estimations. State estimations were treated as optimization issues where SKF agents were Kalman filters. A population agent using a typical Kalman filter framework to solve optimization issues comprised simulated measurement procedures [26]. Their findings from SKF were compared with other metaheuristic algorithms using statistical analysis where findings revealed that the suggested SKF algorithm was a promising technique that outperformed various well-known metaheuristic algorithms such as GAs (Genetic Algorithms), PSOs (Particle Swarm Optimizations), BHAs (Black Hole Algorithms), and GWOs (Grey Wolf Optimizers) [27].

Nonlinear estimators based on KLMSs were proposed by Singh et al. [18], and they outperformed traditional estimators. KLMSs estimators have poor selections of system parameter, and to overcome their limitations, nonlinear estimators, namely, EKFs and UKFs, were used in this study [28]. EKFs were selected due to their ease in implementations, but suffered from inadequate representations of nonlinear functions for 1^st^ order linearization, while UKFs outperformed EKFs by providing stableness by treating nonlinearities precisely. The suggested EKFs- and UKFs-based estimators of the study enhanced accuracies, according to the study's simulation findings [29].

 Eden et al. [30] investigated sub-Nyquist cognitive radars in which overall transmitting powers of multiband cognitive waveforms were conventionally equivalent to full bands which lowered MSEs of single-target TDE estimates. To improve accuracies of delay estimations, the study selected best bands and distributed total power in the bands [31]. Using Cramér–Rao limits, the study showed that, in cognitive radars, equal width subbands resulted in superior delay estimations than conventional radars. Cognitive radars performed effectively in terms of low SNRs in their investigation utilising Ziv-Zakai bounds [32].

Roemer et al. [31] examined challenges in predicting unknown delay(s) as systems receive linear combinations of multiple delayed copies of known broadcast waveforms. This issue was noticed in a variety of applications, including timing-based localizations and wireless synchronizations. With the purpose of reducing hardware complexities, the study suggested compressed sensing-based system design that measured values below Nyquist rates, yet delay estimates were accurate [33]. The study's design of kernels for measurements with frequencies showed optimal numerical choices and outperformed functions that were randomly chosen for estimating delays.

Cobos et al. [29] suggested a subband technique for estimation of TDEs with the goal of increasing traditional GCC (generalized cross-correlation) algorithms. Their suggested method used sliding windows to extract numerous distinct correlations amongst cross-power spectrum's frequency bands of the phase [24]. Their key contributions could be summed up as follows: (1) GCC subband representations of cross-power spectrums which have lower temporal resolutions and estimate TDOAs (time difference of arrival) better; (2) when signals are without noises, their matrix representations exploited scenarios for achieving robust and accurate GCCs; (3) designing low-rank approximations for processing GCC subband matrices resulting in improved TDOA estimates and source localization performances [22]. To show the validity of their suggested technique, their scheme was tested with large number of experiments.

Li et al. [26] introduced a new approach for exploiting space-frequency features to estimate DOAs (direction-of-arrivals) and TDEs of multipath OFDM (orthogonal frequency division multiplexing) signals. The study's scheme combined array structures and frequencies to generate extended virtual arrays. The study reduced impacts of multipath by constructing extended channel frequency response matrices which were smoothened [34]. The study's DOA estimations used quick closed solutions with minimum complications where one-dimensional spectrum searched estimated TDEs. The study's simulations demonstrated that their suggested approaches operated well in a variety of multipath settings, even when SNRs were low. Furthermore, as compared to multidimensional spectral peak search approaches, their methods substantially lowered computing costs with superior estimation performances.

Compressed sensing which reaches high resolutions was exploited by Li and Ma [25] to estimate signal parameters based on the signal's sparseness. Their approaches used high resolutions after l0-norm optimizations. Generalized filter outputs or ambiguous functions result in sparse representations where prior studies used sparse representations for channel responses. The study deconvolved outputs of generalized matching filters using greedy optimizations and Bayesian methods for two-dimensional estimations of Doppler shift and TDEs. Their simulations showed that their technique outperformed other sparse representations of channel data in low SNRs.

## 3. Proposed Methodology

The main aim of this study is to predict TDEs and Doppler shifts (radial velocities) of signals. These estimations are based on nonlinear estimation approaches, namely, multi-iterative function and EKFs. To obtain theoretical optimal solutions, multi-iterative function consumes fewer iterations, resulting in shorter running times, and is useful for estimating target's properties accurately even in complicated contexts. This study's suggested estimators showed lower errors and variances in simulations.

### 3.1. Signal Model Formulation

This section derives radar return signals by connecting radar return and required unknown parameters such as TDEs and Doppler shift where monostatic LFM radars [3] were used to keep radars static.  Figure 1 shows a block diagram of the suggested scheme where monostatic radars were considered. Radars' transmitters emit LFM pulses at baseband frequencies (refer to Figure 1) with LFM pulses separated by set periods called PRIs (pulse repetition intervals). Received signals get dispersed from their initial broadcasting signals. This scattering occurs due to two factors, namely, TDEs (signal transmissions between antennas and targets) and Doppler shifts which occur due to radial velocities of targets.

The LFMSs (v_LFM_(*t*)) can be depicted as

(1) $$\begin{array}{c} v_{\text{LFM}}\left(t\right)=\left\{a\exp\exp\left(j\pi \gamma t^{2}\right)\right.;0\leq t\leq T_{o}\;0;T_{0}<t<T_{\text{PRI}}, \end{array}$$

where *a* represents amplitude, *γ* represents sweep rate's frequency, *T*_*o*_ represents duration of pulses, and T_PRI_ represents PRIs. Frequency of LFMSs varies with time where immediate frequency is computed using *f*_*i*_(*t*)^2^=*γt*. The m^th^ pulse when MLFM pulses burst can be represented as time shift forms of LFMSs and is shown as

(2) $$\begin{array}{c} v_{j}\left(t\right)=v\left(t-nT_{\text{PRI}}\right)for0\leq t\leq T_{o}, \end{array}$$

where *n* ∈ [0,1,…, *N* − 1] and *N* represents total pulse count in a burst. *v*_*j*_(*t*) gets modulated by high-frequency carrier signals where modulations can be represented mathematically as

(3) $$\begin{array}{c} v\left(t\right)=\left\{v_{j}\left(t\right)\right\}\exp\exp\left(j2\pi f_{c}t\right), \end{array}$$

where *f*_*c*_ represents carrier signal's frequency. Returning signals *p*_*m*_(*t*) are time-delayed variants of *v*(*t*), where *τ*_*m*_ stands for TDEs of the m^th^ pulse when equation (4) is satisfied:

(4) $$\begin{array}{c} \tau_{m}=\tau_{o}-\frac{2}{C}\left\{vmT_{\text{PRI}}\right\}, \end{array}$$

where *τ*_*o*_ represents first pulse's TDE, *v* represents radial velocity, and *c* represents light's velocity. For maintaining generality of target's time (*N* pulses), *v* is considered constant or constant Doppler shifts are assumed. Then, time differences 2/*c* {*vm* T_PRI_} in time shifts of return signals when targets change positions over nT_PRI_ result in subsequent changes to *p*_*n*_(*t*) and are given by

(5) $$\begin{array}{c} p_{n}\left(t\right)=\left\{v_{j}\left(t-\tau_{n}\right)\right\}\exp\exp\left(j2\pi f_{c}\left(t-\tau_{n}\right)\right)+k_{m}\left(t\right), \end{array}$$

where *k*_*m*_(*t*) represents additive thermal noises. Returning signals, *p*_*n*_(*t*), of basebands when depicted mathematically take the form

(6) $$\begin{array}{c} p_{m}\left(t\right)=\left\{v_{j}\left(t-\tau_{n}\right)\right\}\exp\exp\left(-j2\pi f_{c}\tau_{n}\right)+k_{m}\left(t\right), \end{array}$$

which implies *P*_*n*_(*f*) can be written as

(7) $$\begin{array}{c} P_{n}\left(f\right)={\left|V_{\text{LFM}}\left(f\right)\right|}^{2}\exp\exp\left(-j2\pi f_{c}\tau_{n}\right)\exp\exp\left(-j2\pi f\tau_{n}\right)+k_{m}\left(f\right), \end{array}$$

where V_LFM_(*f*) represents Fourier transform LFMSs sampling frequency *l*=[0,1,…, *L* − 1] with interval Δ*f*, and dividing by |*V*_LFM_(*l*Δ*f*)|^2^ yields the following equation:

(8) $$\begin{array}{c} p\left(n,l\right)=\exp\exp\left(-j2\pi f_{c}\tau_{n}\right)\exp\exp\left(-j2\pi f\tau_{n}\right)+k\left(n,l\right), \end{array}$$

where *k*(*n*, *l*) represents thermal noise's discrete samples. Substituting *τ*_*n*_ from equation (4) results in the following equation:

(9) $$\begin{array}{c} p\left(n,l\right)=\exp\exp\left(j2\pi nf_{d}T_{\text{PRI}}\right)\exp\exp\left(-j2\pi lf\tau_{o}\right)\exp\exp\left(j2\pi f_{d}ml\left(\frac{T_{\text{PRI}}f}{f_{c}}\right)\right)+k\left(n,l\right), \end{array}$$

where *f*_*c*_= 2vf_c_/*c* represents unknown Doppler shifts caused by target's radial velocities. From equation (9), it can be noted that returning signals, r(m, l), are nonlinearly and exponentially related to TDEs (*τ*_*o*_ and *f*_*d*_) which are estimated from returning signals r(m, l) using EKFs and UKFs. Gaussian filters were used instead of particle filters as they result in acceptable estimation with low processing costs. The suggested EKFs and OIUKFs for estimating TDEs are Gaussian filters. The LFM radar system's state assessment model was developed using Bayesian framework followed by EKFs and OIUKF estimations for *τ*_*o*_ and *f*_*d*_.

This study uses notations for mathematical representations where constants are in uppercases, vectors are boldfaced uppercases, superscript representations are ^T^transposes, ^H^complex conjugate transposes of matrices, and ^*∗*^scalar complex conjugate operations, statistical expected outcomes are represented by *E*[*·*], and *R* denotes real numbers, while *C* stands for complex numbers where *R* (·) implies real parts and *I* (·) stands for imaginary parts.

### 3.2. State Assessment Models for RSs

The suggested state evaluations in this study contain measurement models in which the states are assessed via the use of mathematical linkages. The state is represented by the TDEs (_o and *f d*), whilst the observed values (returning signals *p*(*n*,*l*)) are represented by the measurements and variables specified as *x* = [ *o f d*]*T* and *y* = [*R*(*r*(*m*,*l*))*I*(*r*(*m*,*l*))]*T*, respectively. Because of the expected stability of radial velocities in the state space model specified in equation (9), the intervals and TDEs in the model grow consistently. The errors resulting from the constant assumptions used in this research are referred to as process noise.

The modelled state can be depicted mathematically as

(10) $$\begin{array}{c} y_{k+1}=f\left(y_{k}\right)+\eta_{k}=y_{k}+\Delta y+\eta_{k}, \end{array}$$

where *k* ∈ {1,2,…, *K*}, *K*=ML stands for discretized sample counts of signals returned, and Δ*x*=[*T*_*o*_/*K*, 0] represents changes/shifts between successive returning signals. *η*_*k*_ represents noises that are additive and assist in modelling error compensations. Based on equation (9), measurements (*x*_*k*+1_) can be depicted as

(11) $$\begin{array}{c} x_{k+1}=c\left(x_{k+1}\right)+d_{k+1}\\ =\left[\begin{array}{c} R\left(\exp\exp\left(j2\pi ny_{k+1}\left(2\right)T_{\text{PRI}}\right)\exp\exp\left(-j2\pi l\Delta fy_{k+1}\left(1\right)\right)\exp\exp\left(j2\pi y_{k+1}\left(2\right)ml\left(\frac{T_{\text{PRI}}\Delta f}{f_{c}}\right)\right)\right)\\ I\left(\exp\exp\left(j2\pi ny_{k+1}\left(2\right)T_{\text{PRI}}\right)\exp\exp\left(-j2\pi l\Delta fy_{k+1}\left(1\right)\right)\exp\exp\left(j2\pi y_{k+1}\left(2\right)ml\left(\frac{T_{\text{PRI}}\Delta f}{f_{c}}\right)\right)\right) \end{array}\right]\\ +v_{k+1}, \end{array}$$

where *d*_k_ stands for noises measured. These measurements help mitigate signal errors that occur while collecting/processing them. *η*_*k*_ and *v*_*k*_ represent Gaussian filter's assumed zero means with covariance *Q*_*k*_ and *R*_*k*_ This study considers additive impacts of process/measurement noises.

### 3.3. Bayesian Filters

Bayesian filtering is two-step operations using predictions and updates.

#### 3.3.1. Predictions

This phase creates the PDFs (probability distribution functions) of state one-time step forward (relation to the available observations) by utilising Chapman–Kolmogorov equation [35] given as follows:

(12) $$\begin{array}{c} P\left(x_{1:k-1}\right)=\int P\left(y_{k-1}\right)P\left(x_{1:k-1}\right)\text{d}y_{k-1}, \end{array}$$

where P(·) stands for PDFs and *P*(*x*_1:*k*−1_) stands for prior PDFs.

#### 3.3.2. Update

PDFs are reconstructed in this step when new measurement values from Bayes rule [35] *y*_*k*_ are received and depicted as

(13) $$\begin{array}{c} P\left(y_{1:k-1}\right)=P\left(y_{1:k-1},y_{k}\right)=\frac{1}{c_{k}P\left(x_{k}\right)P\left(y_{1:k-1}\right)}, \end{array}$$

(14) $$\begin{array}{c} c_{k}=P\left(y_{1:k-1}\right)=\int P\left(x_{k}\right)P\left(y_{1:k-1}\right)\text{d}x_{k}, \end{array}$$

where *P*(*x*_*k*_) stands for likely measures achieved using equation (11) and *c*_k_ represents constant for normalizations. The use of Bayesian filtering results in the construction of posterior PDFs *P*(*y*_1:*k*_).

### 3.4. TDE Estimations Using EKFs

The estimations of TDEs (*τ*_*o*_ and *f*_*d*_) from returning signals, *r*(*m*, *l*), of the investigated RSs using equations (10) and (11) are simplified from state assessment as estimations of *x k* from known *y k* measurements where EKFs are analytical simplifications of Bayesian frameworks and conditional PDFs in Bayesian framework equations (12)–(14) are assumed to be Gaussians as shown in the following equations:

(15) $$\begin{array}{c} P\left(x_{k|k-1}\right)∼N\left(x_{k|k-1};{\hat{x}}_{k|k-1},P_{k|k-1}\right), \end{array}$$

(16) $$\begin{array}{c} P\left(x_{k|k}\right)∼N\left(x_{k|k};{\hat{x}}_{k|k},P_{k|k}\right), \end{array}$$

where real Gaussian distributions are represented as *N*. *x*_*k|k*−1_ stands for mean values, while *P*_*k|k*−1_ implies covariance of *x*_*k|k*−1_ and similarly *x*_*k|k*_ implies mean values and *P*_*k|k*_ covariance of *x*_*k|k*_. *x*_*k|k*−1_ and *P*_*k|k*−1_ are predicted, while *x*_*k|k*_ and *P*_*k|k*_ are updated as detailed below.

#### 3.4.1. Prediction

In this step, prior PDFs (*x*_*k|k*−1_ and *P*_*k|k*−1_) result when Jacobian (*F*_k_) of *f*(*x*_*k*_)  [35] is used and depicted as follows:

(17) $$\begin{array}{c} F_{k}=\frac{\partial f\left(x\right)}{\partial x}|x={\hat{x}}_{k-1|k-1}=\left[1001\;\right]. \end{array}$$

#### 3.4.2. Update

In the initial part of this step, measurements $\left({\hat{y}}_{k|k-1}\right)$ are predicted along with error covariance (*P*_*k|k*−1_^YY^) using Jacobian (*H*_k_) of h(·) [35] which results in new measurements *y*_*k*_. Subsequently, posterior estimates and covariances, ${\hat{x}}_{k|k-1}$ and *P*_*k|k*_, are obtained using Kalman filter gains (*K*_*k*_) where posterior estimations ${\hat{x}}_{k|k}={\left[{\hat{\tau }}_{o_{k}}{\hat{f}}_{d_{k}}\right]}^{T}$ result desired TDEs and Doppler shift outcomes.

### 3.5. Optimized Iterative Unscented Kalman Filter (OIUKF)

The calculation of an IUKF using the Fisher estimation framework is described in [36], and it entails minimizing the following cost function in the filter's measurement update phase:

(18) $$\begin{array}{c} {\hat{y}}_{t|t}=Z\left(y\right)=\frac{1}{2}f^{T}\left(y\right)f\left(y\right), \end{array}$$

(19) $$\begin{array}{c} f\left(y\right)=\left[R_{t}^{-1/2}\left(y_{t}-h\left(x\right)\right)P_{t|t-1}^{-1/2}\left({\hat{x}}_{t|t-1}-x\right)\right], \end{array}$$

(20) $$\begin{array}{c} H_{i}={\left(P_{i}^{xy}\right)}^{T}P^{-1}. \end{array}$$

It presupposes, like the IUKF version, that the measurement function is affine in the vicinity of *x* and *x i* and therefore that *h*_*x*_' (*x*) = *h*_x_' (*x*_i_) = *H*_*i*_. The Jacobian *H*_*i*_ is not explicitly computed in the UKFs, but the fact that *P*^*xy*^ = *P*^HT^ in the linear case may be used to infer a stochastic linearization. As a result, the equation provides a fair estimate of *H*_*i*_ in the IUKF (20).

When P's symmetry has been exploited, *P*^*xy*^ implicitly incorporates second-order transformation effects [37]. The state iteration in IUKF may be utilised to generate the following equation using the preceding stochastic linearization approach:

(21) $$\begin{array}{c} x_{i+1}=\hat{x}+K_{i}\left(y-{\hat{y}}_{i}-{\left(P_{i}^{xy}\right)}^{T}P^{-1}\left(\hat{x}-x_{i}\right)\right), \end{array}$$

(22) $$\begin{array}{c} K_{i}=P_{i}^{xy}{\left(P_{i}^{yy}\right)}^{-1}, \end{array}$$

(23) $$\begin{array}{c} {\hat{y}}_{i}=\sum_{k}W^{\left(k\right)}Y_{i}^{\left(k\right)}. \end{array}$$

It can be utilised as a starting point in the IUKF. It is worth noting that *y*  = *y* (*t*|*t*-1) remains constant. The projected measurement *y* i must still be determined. The following equation can be used to express two different natural alternatives:

(24) $$\begin{array}{c} {\hat{y}}_{i}^{*}=Y_{i}^{\left(0\right)}, \end{array}$$

i.e., the converted centre sigma point, represented by the superscript ^*∗*^ in this case. Two somewhat different interpretations of the cost function by equation result from the options (25) and (26):

(25) $$\begin{array}{c} V\left(x\right)={\left(y_{t}-E\left[h\left(x\right)\right]\right)}^{T}R_{t}^{-1}\left(y_{t}-E\left[h\left(x\right)\right]\right)+{\left({\hat{x}}_{t|t-1}-x\right)}^{T}P_{\left(t-1\right)}^{-1}\left({\hat{x}}_{t|t-1}-x\right), \end{array}$$

(26) $$\begin{array}{c} V^{*}\left(x\right)={\left(y_{t}-h\left(x\right)\right)}^{T}R_{t}^{-1}\left(y_{t}-h\left(x\right)\right)+{\left({\hat{x}}_{t|t-1}-x\right)}^{T}P_{\left(t-1\right)}^{-1}\left({\hat{x}}_{t|t-1}-x\right), \end{array}$$

both depict different approximations of costs where corrections to states can result in decreased costs, i.e., *V*(*x*_*i*+1_) < *V*(*x*_*i*_). If this is not the case, a step size parameter *α* is given by

(27) $$\begin{array}{c} y_{j+1}=y_{j}+\alpha_{j}\left(\hat{y}-y_{j}+G_{j}\left(x-{\hat{x}}_{j}-H_{i}\left(\hat{x}-x_{i}\right)\right)\right). \end{array}$$

MCEHOs are used to compute the step sizes where EHOs (Elephant Herding Optimizations) use both global and local searches [38]. Local searches, on the other hand, aim to locate better step sizes in smaller search spaces with smaller promising approximate predictions of time and Doppler flaws. Elephant's herding behaviours are characterized as elephant populations (with varying step sizes) split into clans. Generations have males which leave their clans for optimal selections of step sizes. Clans represent local searches in the algorithm through the optimum selection of step sizes, but male elephants leaving clans are global search implementations through step sizes. Matriarchs are solution (elephants) in the clan with the best fitness values for TDEs. Moving male elephants, on the other hand, are solutions *τ*_*o*_ and *f*_*d*_ with the worst fitness function of RSs. MCEHO approach divides elephant population into *k* clans, which are D-dimensional solutions created randomly in search spaces by using lower bounds *x*_*min*_ and upper bounds *x*_*max*_ of TDEs and using

(28) $$\begin{array}{c} x=x_{\min}+\left(x_{\max}-x_{\min}+1\right)r\mathrm{and}, \end{array}$$

where rand implies random numbers between 0 and 1. New solutions get generated in generations when clan members (*j*) from clan (*c*_*i*_) with best fitness values get attracted by solutions (*x*_*best*,*c*_*i*__) [38]:

(29) $$\begin{array}{c} x_{\mathrm{new},c_{i},c_{j}}=x_{c_{i},c_{j}}+\alpha_{\mathrm{mutation}}\left(x_{\mathrm{best},c_{i}}-x_{c_{i,j}}\right)rand, \end{array}$$

where *x*_new,*c*_*i*_,*c*_*j*__ represents *j*'s new solution in clan *c*_*i*_ for optimal selection of steps size in TDEs and Doppler effects, *x*_*c*_*i*_,*c*_*j*__ represents previous generation's solution, *α*_mutation_ represents generated parameter via mutation operator, and algorithm's parameter is set correspondingly for TDEs and Doppler effect. If the mutated value is worse than the new value that is created via new mutated value, *rand* ∈ [0,1] random numbers between (0,1) in uniform distributions. Scaling factor *α* influences best TDEs and Doppler effect values with their step sizes. and these positions in clans get updated based on the equation [38] given below:

(30) $$\begin{array}{c} x_{\mathrm{new},c_{i}}=\beta x_{\mathrm{center},c_{i}}, \end{array}$$

where [0, 1] is the second algorithm parameter, which determines the clan centre's effect, *x*_*center*,*c*_*i*__, for TDEs and Doppler effect. Clan centre is defined by the following equation [38]:

(31) $$\begin{array}{c} x_{\mathrm{center},c_{i,d}}=\frac{1}{n_{c_{i}}}\sum_{l=1}^{n_{c_{i}}}x_{c_{i,l,d}}, \end{array}$$

where 1 ≤ *d* ≤ *D* represents the *d*^th^ dimension and *n*_*c*_*i*__ is the number of reduced TDEs and Doppler effect in clan *c*_*i*_. In each clan, *n*_*c*_*i*__ solutions with the worst fitness values for TDEs and Doppler effect of the clan *c*_*i*_ are chosen to be replaced by the following equation [39]:

(32) $$\begin{array}{c} x_{\mathrm{worst},c_{i}}=x_{\min}+\alpha \left(x_{\max}-x_{\min}+1\right)\mathrm{rand}, \end{array}$$

where *x*_*min*_ and *x*_*max*_ represent lower and upper bounds of search spaces for TDEs and Doppler effects in the interval rand∈[0, 1]. TDEs and the Doppler effect were used to represent a random integer from uniform distributions where they use two separate one-dimensional maps, circles, and sinusoidal maps to generate random numbers [40]. The circular maps [39] can be described by

(33) $$\begin{array}{c} y_{g+1}=\left[y_{g}+a-\frac{b}{2\pi }\sin\sin\left(2\pi y_{g}\right)\right]\mathrm{mod}1, \end{array}$$

where the produced chaotic sequence is inside *b* = 0.5 and *a* = 0.2 (0, 1). The equation for a sinusoidal map is as follows [39]:

(34) $$\begin{array}{c} y_{g+1}=by_{g}^{2}\sin\left(\pi y_{g}\right), \end{array}$$

where for *b* = 2.3 and *y*_0_ = 0.7, the following simplified form is obtained.

## 4. Results and Discussion

The proposed scheme using EKFs and OIUKF estimations were tested with MATLAB simulations and compared with other nonlinear estimators based on UKFs, KLMSs, and modified NCs. Two monostatic ECG with different parameter values were studied and are listed in Table 1 for scenarios 1 and 2, which refer to the two ECG [34]. Scenario 1 depicts realistic LFM ECG, where parameter values differ from those of Scenario 2's ECG.

For both scenarios 1 and 2 estimators based on EKFs and multi-iterative function, *R*_k_ = *σ*^2^I (where *σ*^2^ is obtained according to specified SNRs defined as relative strengths of signals with respect to noises in this work).

(35) $$\begin{array}{c} \text{SNR}=h{\left(x_{k+1}\right)}^{T}\frac{h\left(x_{k+1}\right)}{n\sigma^{2}}. \end{array}$$

TDEs and Doppler shift were estimated for SNR of 20 dB; however, a comparative study is presented for SNRs ranging from 30 dB to 20 dB. The proposed algorithm of both scenarios sigma=0.5 was evaluated with and 5 sigma points in simulations taking 2n +1 (where *n* is the dimension or 2 in this study).

Using EKFs and OIUKF-based estimating procedures, the final NMSE can be achieved after approximately three thousand and fifty-five iterations, UKFs-based estimation can be achieved after approximately three thousand and fifty-five iterations, and KLMS-modified NC can be achieved after approximately four thousand and fifty-five iterations. Furthermore, compared to the other techniques, OIUKF produces a much lower end NMSE than the others. The OIUKF estimator converges rapidly and produces much lower final MSE than earlier techniques, in contrast to estimators based on EKFs, UKFs, and KLMS-modified NC, which need longer time to converge. As shown in Figure 2, for 5000 iterations in scenario 1 in estimation of TDEs, the proposed OIUKF-based estimation has a lower mean square error (NMSE) of 0.0032, whereas other approaches such as EKFs, UKFs, and KLMS-modified NC have higher mean square errors (NMSEs) of 0.42, 0.029, and 0.012, respectively.  Figure 3 represents the 5000 iterations in the proposed work.

Table 2 represents the noise estimation of the proposed work.

In Doppler shift estimation, the proposed OIUKF-based estimation yields a decreased NMSE value of 0.00094, whereas other approaches such as EKFs, UKFs, and KLMS-modified NC give higher NMSE values of 0.36, 0.045, and 0.0092, respectively, after 5000 iterations in scenario 2 represented in Figure 4.

Figure 4 shows that the proposed OIUKF-based estimation has a lower NMSE of 0.00092, whereas other approaches such as EKFs, UKFs, and KLMS-modified NC have higher NMSEs of 0.33, 0.020, and 0.0087, respectively, after 5000 iterations in scenario 2 in estimation of TDEs.

## 5. Conclusion and Future Work

TDEs and Doppler shifts are used in ECG to derive measures such as ranges and radial velocities. The proposed multi-iterative function and the EKFs are two unique nonlinear estimation approaches that can overcome estimator's limitations, with enhanced outcomes for TDEs and Doppler shifts. Nonlinearity is regarded as the genuine nonlinear model for estimation in the proposed OIUKF system. MCEHOs are used to optimise a new parameter using a cost function. The OIUKF system uses numerical approximation to provide a derivative-free implementation. It is more stable than the EKFs since it is implemented without derivatives. EKFs are favorable because of their ease in implementations, but they suffer from inadequate representations of nonlinear functions by first-order linearization, whereas the proposed multi-iterative function outperforms EKFs while having better stability due to precise treatment of system's nonlinearity. As a result, the multi-iterative function outperforms EKFs in terms of stability and yield estimates that are better/similar in accuracies. In actuality, however, clutter, which is frequently represented as non-Gaussianity, is common. As a result, the nonlinear form of the Kalman filter capable of coping with non-Gaussianity can be researched in the future to deal with the impacts of clutter. The tracker also requires range, radial velocity, and angle information for accurate tracking.

## Figures and Tables

**Figure 1:** Block diagram of the proposed ECG.

**Figure 2:** For scenario 1, NMSE plots of time delay estimation with estimators based on KLMS-modified NC, UKFs, EKFs, and OIUKF.

**Figure 3:** NMSE plots of Doppler shift estimation for scenario 1 using estimators based on KLMS-modified NC, UKFs, EKFs, and OIUKF.

**Figure 4:** For scenario 2, NMSE plots of time delay estimation with estimators based on KLMS-modified NC, UKFs, EKFs, and OIUKF.

**Algorithm 1:** Pseudocode of the MCEHO algorithm.

**Table 1:** LFM radar values of scenario I and scenario II used for simulation.

S.N.	Quantity	Values for scenario 1	Values for scenario 2
1	Number of pulses (M)	10	20
2	Number of frequency intervals (L)	500	500
3	Frequency increment (∆f)	10 MHz	10 MHz
4	Pulse duration (T0)	5 us	200 us
5	Pulse repetition interval (Tpri)	1 ms	0.4 ms
6	Centre frequency (fc)	10 GHz	9 GHz

Modified NCs. Two monostatic ECG with different parameter values were studied and are listed in Table 1 for scenarios 1 and 2, which refer to the two ECG [34]. Scenario 1 depicts realistic LFM ECG, where parameter values differ from those of scenario 2's ECG.

**Table 2:** NMSE estimation values of scenario I for estimators.

No. of iterations (*k*)	Time delay estimation				Doppler shift estimation			
	KLMS-modified NC	EKF	UKF	OIUKF	KLMS-modified NC	EKF	UKF	OIUKF
1000	1.28	0.095	0.044	0.0091	0.97	0.095	0.044	0.0082
2000	1.12	0.082	0.036	0.0067	0.68	0.072	0.026	0.0064
3000	0.98	0.055	0.022	0.0054	0.51	0.064	0.022	0.0042
4000	0.67	0.045	0.015	0.0046	0.43	0.051	0.015	0.0026
5000	0.42	0.029	0.012	0.0032	0.36	0.045	0.0092	0.00094

## Data Availability

The data that support the findings of this study are available on request to the corresponding author.
